# The Oncolytic Virus in Cancer Diagnosis and Treatment

This article has been retracted.

**DOI:** 10.3389/fonc.2020.01786

**Published:** 2020-09-09

**Authors:** Guo-dong Cao, Xiao-bo He, Qiang Sun, Sihan Chen, Ke Wan, Xin Xu, Xudong Feng, Peng-ping Li, Bo Chen, Mao-ming Xiong

**Affiliations:** ^1^Department of General Surgery, The First Affiliated Hospital of Anhui Medical University, Hefei, China; ^2^Jiangsu Key Laboratory of Biological Cancer, Cancer Institute, Xuzhou Medical University, Xuzhou, China; ^3^Department of Oncology, Anhui Medical University, Hefei, China; ^4^Department of Infectious Disease, Zhejiang University, Hangzhou, China; ^5^Department of General Surgery, The First People’s Hospital of Xiaoshan District, Hangzhou, China

**Keywords:** cancer, oncolytic virus, application, review, diagnosis

## Abstract

Cancer has always been an enormous threat to human health and survival. Surgery, radiotherapy, and chemotherapy could improve the survival of cancer patients, but most patients with advanced cancer usually have a poor survival or could not afford the high cost of chemotherapy. The emergence of oncolytic viruses provided a new strategy for us to alleviate or even cure malignant tumors. An oncolytic virus can be described as a genetically engineered or naturally existing virus that can selectively replicate in cancer cells and then kill them without damaging the healthy cells. There have been many kinds of oncolytic viruses, such as herpes simplex virus, adenovirus, and Coxsackievirus. Moreover, they have different clinical applications in cancer treatment. This review focused on the clinical application of oncolytic virus and predicted the prospect by analyzing the advantages and disadvantages of oncolytic virotherapy.

## Introduction

Malignant tumors killed over 8 million people worldwide in 2013 and have moved from the third leading cause of death in 1990 to the second leading cause behind cardiovascular diseases in 2013 (1, 2). In China, the incidence and mortality of cancer are increasing year by year. According to relevant data, the mortality rate of Chinese residents with malignant tumors has increased by 83.1% since the mid-1970s (3). Malignant tumors have become one of the leading causes of death all over the world. Although there are already many treatments including surgical treatment, radiotherapy, chemotherapy, and the latest immunotherapy that can prolong the survival period of tumor patients, they have some limitations. Surgical treatment is mainly used for early stage cancer patients, while severe side effects make radiotherapy and chemotherapy hard for patients to tolerate. Besides, traditional immunotherapy still has many defects; for example, the objective effectiveness of patients receiving immunotherapy is only 10 to 30%, so improving the efficiency of immunotherapy is urgently needed (4). Comprehensively, existing cancer treatment strategies are imperfect, and new treatment methods need to be proposed that should have accurate tumor targeting, powerful tumor-killing properties, and low toxic side effects.

Oncolytic virotherapy is a treatment of using a virus that can replicate itself to kill cancer cells. There are many species of viruses, but not all of them can be designed to be an oncolytic virus (OV) (5). The typical features of these OVs must include being non-pathogenic, the ability to target and kill the cancer cells, and the capacity of being transformed to express tumor-killing factors through genetic engineering methods (6). Tumor selectivity could be concerned with the level of receptor-mediated cell entry, intracellular antiviral responses, or restriction factors that determine the susceptibility of the infected cell that leads to viral gene expression and replication (7, 8). The history of treating cancer with microbes dates back to 1890; a surgeon named William B. Coley in the Memorial Hospital in New York was the first to observe the regression of tumors in several patients infected with the pathogen. Moreover, he called the pathogen antitumor agents (9, 10). In 1935, *Clostridium histolyticum* was used by Connell to treat advanced cancers, and tumor regression was observed not long after that (11). Later, in the 1950–1970s, live viruses were deliberately injected into cancer patients and showed positive activity, such as Egypt 101 West Nile virus (4/34 transient regressions), adenovirus lysates (26/40 showing localized tumor necrosis), and Urabe strain mumps virus (37/90 complete remission or partial responses) (9). However, some side effects were emerging in these early researches by using natural viruses, because these viruses were not engineered for tumor selectivity, especially in immunosuppressed patients with leukemia or lymphoma (five of eight patients had severe encephalitis after being treated with West Nile virus) (9, 12).

The OV has become a promising treatment to fight cancer in the new era. It is reasonable to believe that oncolytic virotherapy has the potential to become one of the primary therapies to treat cancer. The emergence of oncolytic virotherapy not only revolutionizes the standard of cancer treatment but also innovates the concept of cancer treatment. It is called the third revolution of tumor treatment after traditional chemotherapy and targeting therapy. The primary purpose of this review is to present the latest advances in clinical applications or trials of various OVs and to look forward to the future based on the current shortcomings of OVs.

## The Origin and Development of Oncolytic Virus Treatment

The concept of using viruses to treat tumors has been around for more than 100 years. As early as 1904, a 42-year-old woman with leukemia was reported to have had her tumor receded due to influenza. Then, in 1912, Italian doctors found that rabies vaccine injection can cause cervical cancer regression, which led to the emerging concept of OV therapy and a series of related studies (13). In the 1950s and 1970s, the researchers conducted a lot of clinical trials using wild-type viruses for the treatment of tumors, but due to the inability to effectively control the pathogenicity of the virus, the OV settled at the second place in cancer therapies. It was not until the 1980s that the emergence of genetic engineering technology made it possible to modify the genome of a virus, followed by the emergence of genetically engineered attenuated and highly selective viruses. In 1991, preclinical animal experiments reported that the gene-modified human herpes simplex virus I (HSV-1) by knocking out thymidine kinase (TK) could inhibit the growth of glioma in mice, prolong the survival of mice, and have excellent safety. In 1996, onyx-015, a genetically modified adenovirus, entered phase I clinical trials (14, 15). In 2004, RIGVIR, a non-pathogenic enteric cytopathic human orphan virus, was approved in Latvia for the treatment of melanoma and became the first OV approved by regulatory authorities for cancer treatment. In 2005, the modified adenovirus H101 (Oncorine, recombinant human adenovirus five injection, ankeri) was approved in China, but its clinical efficacy has not been internationally recognized (16). In October 2015, the Food and Drug Administration (FDA) approved the marketing of T-VEC (talimogene laherparepvec, Imlygic). In 2016, T-VEC was approved to market in Europe and Canada, marking the maturity of OV technology for the treatment of cancer. Currently, three OV products have been approved for marketing, and six more OV products are in phase III clinical studies (17). Compared with other tumor immunotherapies, OVs have many advantages, such as high killing efficiency, precise targeting, fewer side effects or drug resistance, and low cost (18). All of these make oncolytic virotherapy a promising therapy to fight cancer compared with surgical therapy, chemoradiotherapy, and targeted therapy.

The OV contains a wide range of viruses that have some common characteristics that virotherapy relies on. Malignant cells are more susceptible to OV infection because of the specific cytokines they expressed. On the one hand, it is reported that tumor-driver mutations enhance the selectivity of viruses in cancer cells (19, 20). Furthermore, many tumor cells supported the replication of selective viruses, maybe because of the lack of antiviral type I interferon signaling (21). In addition to this part, the size and complexity of different OVs are diverse, such as vaccinia [190 kilobases (kb)] and HSV1 (152 kb) to the tiny parvovirus H1 (5-kb linear, single-stranded DNA) (22, 23), which may lead to differences in the ability of the virus to infect tumor cells.

## The Application of Oncolytic Virus

Three viruses currently in clinical use, RIGVIR, Oncorine, and T-VEC, have shown satisfactory therapeutic effects. Besides, many OVs are in preclinical trials; among them, herpesvirus, adenovirus, and vaccinia virus presented good experimental results. Below, we will describe the application of different OVs in tumor diagnosis and tumor treatment.

### Cancer Diagnosis

At present, all kinds of advanced imaging technology for the diagnosis of tumor play an irreplaceable role, especially CT and MRI, in the accurate positioning and local invasion assessment of tumor. However, the early detection of primary tumors and small metastases still cannot be effectively acquired, so higher sensitivity and accuracy of imaging technology need to be discovered. In recent years, accurate tumor imaging using OV has attracted more and more attention. OVs with specific genes can selectively infect tumor cells and replicate within them or express genes of interest such as luciferase reporter gene and human Na+/I- symporter (hNIS) gene (24), and we can detect gene expression products such as fluorescence in cancer cells to obtain non-invasive real-time molecular imaging *in vivo* (25). Fluorescence imaging was also one of OVs’ applications in tumor precise imaging. Generating from invertebrate marine animals, the green fluorescent protein (GFP) can be utilized to detect tumor behaviors, including amplification, invasion, and metastasis. In a study by Rojas JJ, the mouse models expressed GFP successfully after injection of adenovirus, vesicular stomatitis virus (VSV), vaccinia virus, and measles virus with GFP gene as compared with other imaging technologies (26). The result showed that tumor imaging with the OV had significantly higher accuracy and agility. Besides, the OV also showed unique advantages in nuclear medical imaging. The reporter genes expressed by the OV in cancer cells can be detected by nuclear medical equipment to acquire the precise location of tumor sites. The current commonly used reporter genes include human sodium–iodine symporter gene (*hNIS*), TK gene, and human type 2 somatostatin receptor gene (*hSSTR2*). Moreover, they all showed good results in mouse model trials or clinical trials (27–30). Imaging techniques commonly used to detect tumors with OVs include optical molecular imaging (bioluminescence imaging and fluorescence imaging), single-photon emission CT (SPECT)/CT, PET, and MRI. All of the above may facilitate the assessment of safety and treatment efficacy of oncolytic virotherapy, as well as a more specific diagnostic technique to detect tumor origin (31,32). So OVs have unique advantages in precise imaging of tumor tissues, and the combination of OVs and imaging methods has great potential in early stage tumor diagnosis. Details are listed in Table 1 (33–37).

**TABLE 1:** The application of oncolytic virus for cancer diagnosis.

Imaging techniques	Cancer	Viruses	Genes	Results
Bioluminescence imaging (27)	Breast cancer	Herpes simplex virus, Herpes simplex virus-1, Herpes simplex virus-Luc	Luciferase	Viral replication cycles can be monitored by bioluminescence imaging
Fluorescence imaging (28)	Breast cancer	Vaccinia virus, Lister strain GLV 1h153	Green fluorescent protein	All positive surgical margins can be observed through FI by the infection of GLV-1h153
SPECT/CT (29)	Prostate cancer	Adenovirus serotype, adenovirus serotype 5, adenovirus serotype 5-yCD/mutTKSR3 9rep-hNIS	Human Na+/I- symporter gene	Tumor imaging was detected in seven of nine (78%) patients
PET (30)	Gastric cancer	Vaccinia virus, Lister strain, GLV-1h153	Human Na+/I- symporter gene	Tumor imaging can be visualized through 99mTc pertechnetate SPECT and 124I PET by the infection of hNIS expressing GLV-1h153
MRI (31)	Prostate tumor	Vaccinia virus, Lister strain, GLV-1h68, GLV-1h312, GLV-1h460, GLV-1h462	Tyrosinase, Tyrosinase p1, Tyrosinase p2, Melanin	The tumor signal enhancement of MRI can be detected after infection of GLV-1h462. The expression of melanin can be controlled by the doxycycline inducible promoter-system and thereby decrease inhibition of viral replication due to melanin overproduction

*GLV, green fluorescent protein-expressing vaccinia virus.*

### Cancer Treatment

The three oncolytic viral drugs currently approved for some clinical cancer treatment are RIGVIR, Oncorine, and T-VEC, and they all have achieved good therapeutic effects. Details are listed in Table 2. And the current clinical trials of OV are shown in Tables 3, 4.

**TABLE 2:** The application of oncolytic virus for cancer treatment.

	Time to market	Virus type	Range of application	Efficacy	Side effects
RIGVIR	2004	Human intestinal cytopathic orphan virus	Melanoma	Among melanoma patients, the overall rate (3-year and 5-year) of rigvir patients and control were 78–84%, 66–81% and 54–57%, 42–56%	Fatigue, sleepiness, and dyspepsia (reversible, lasted for a couple of days and did not require treatment)
Oncorine	2005	Adenovirus	Head and neck cancer	Oncorine plus chemotherapy-treated head and neck cancer patients (78.8%) have a significantly higher response rate compared with the chemotherapy-treated head and neck cancer patients (39.6%)	Fever (45.7%), local site pain (28.3%), flu-like symptoms (9.8%), leukopenia, decreasing platelets, liver malfunctions, alopecia and nausea (all of which were tolerated well)
0.T-vec	2015	Herpes simplex virus	Local treatment of unresectable lesions of recurrent melanoma after surgical excision	Treat advanced melanoma. The overall response rate was 26%. The combined use of T-vec and PD-1 showed a tumor remission rate as high as 62%, of which 33% was complete remission. The remission rate of T-vec alone is 30% to 40%	Chills, fever, injection point pain, nausea, flu-like symptoms, and fatigue. And the most common serious side effects were disease progression, cellulitis, and fever, none of which occurred in more than 2% of cases

**TABLE 3:** The clinical trials of oncolytic virus from published literature.

	Range of trials	Efficacy	Side effects
Vaccinia Virus	Liver cancer	Increased survival of patients with liver cancer after intravenous injection	Flu-like symptoms and Local symptoms
Coxsackievirus	Advanced melanoma	The preliminary durable response rate was 21% with regression of distant lesions	Mild flu-like symptoms, which may be more severe after systemic administration, and local reaction at the injection site
Polio Virus	Glioblastoma	PVS-RIPO showed durable radiographic and clinical responses in glioblastoma	Mild flu-like symptoms, which may be more severe after systemic administration, and local reaction at the injection site
Retrovirus	Malignant glioma	Converts 5-fluorocytosine to the toxic metabolite 5-fluorouracil. And Toca 511 is in a phase 2/3 clinical trial for malignant glioma and has shown promising effects	Mild flu-like symptoms, which may be more severe after systemic administration, and local reaction at the injection site
Parvovirus H1	Pancreatic cancer	Wild-type parvovirus H1-ParvOryx is currently in trials for metastatic pancreatic cancer and has shown promising results	Mild flu-like symptoms, which may be more severe after systemic administration, and local reaction at the injection site
Vesicular Stomatitis Virus	Liver cancer	An engineered VSV that overexpress interferon β is currently in a clinical trial for liver cancer	Mild flu-like symptoms, which may be more severe after systemic administration, and local reaction at the injection site

**TABLE 4:** The clinical trials of oncolytic virus from www.clinicaltrials.gov.

Oncolytic virus	Study type	Condition	Enrollment	Results
HF10	Innervational	Resectable Stage IIIB, IIIC, IVM1a melanoma	7	HF10 was used in combination with Nivolumab to treat melanoma patients in this clinical trial. The overall survival of patients was about 2 years and the pathologic complete response was 83.3% (a pathologic complete response was defined as no viable residual melanoma cells in the surgical specimen)
Oncolytic measles virus	Innervational	Ovarian cancer or primary peritoneal cavity cancer	37	27 of the 37 ovarian cancer or primary peritoneal cavity cancer patients achieved SD (stable disease) for 1 year
Coxsackievirus A21	Innervational	Stage IIIc and stage IV malignant melanoma	57	Percentage of participants with Immune-related progression-free survival (irPFS) at 6 months was 38.6% and the duration response rate was 21.1%
T-vec	Innervational	Stage IIIc and stage IV malignant melanoma	50	The objective tumor response rate of the participants was 28%. The duration of response was 223 days and the overall survival was 448 days

#### Rigvir

Riga virus is an inartificial Enteric Cytopathogenic Human Orphan type 7 (ECHO-7) picornavirus that has been approved for the treatment of melanoma in Latvia, Georgia, and Armenia so far. At the same time, it became the first OV that obtained regulatory approval all around the world in 2004 (38). Although it has gained regulatory approval, there are few articles to describe its biological characteristics and efficacy when used in the treatment of malignant tumors. Only three English-language articles relating to Rigvir are publicly available, including one review article, one case study on three patients, and one retrospective analysis of early stage melanoma patients (38–40). Among them, the retrospective research found that early stage melanoma patients (IB, IIA, IIB, and IIC) who received surgical resection and Rigvir (*n* = 52) survived longer than patients who received surgical resection alone (*n* = 27). Though all patients were pronounced disease-free following surgery, Rigvir was administered post-surgery only after the surgical wounds had healed. Low-grade melanomas after surgical resection seemed to be more sensitive to the treatment of Rigvir. However, the potential of Rigvir to treat high-grade melanoma patients remains unknown, because the English-language reports only contain case studies without more extensive trials (39). However, we believe that as we learn more about the mechanism of how Rigvir works to fight cancer, better treatments for malignancies will be on the horizon.

#### Oncorine (H101)

Oncorine not only was the first approved OV for clinical use in China but also is the world’s first recombinant OV (40). It was applied for the treatment of patients with head and neck cancer after being approved by the Chinese State FDA (SFDA) in 2005 (41). Oncorine is an attenuated serotype five adenoviral vector with a deletion in viral E1B-55k and four deletions in viral E3. As a robust p53 repressor, there was a hypothesis that E1B-55k plays an essential role in the selective replication of Oncorine in p53-deficient tumors. E1B-55k can inhibit the apoptosis of infected cells and allows viral replication in p53-positive cells (42). However, another mechanism of cancer’s selectivity may exist for the fact that E1B-55k-deleted adenoviruses have been proved to infect and replicate in p53-positive tumors (43–45). P14ARF and YB-1 may play a role in an RNA export-dependent mechanism of tumor selectivity (46). After a variety of comprehensive and randomized trials, researchers began to carry out the clinical testing of Oncorine. The operation method was that patients received combination cisplatin and 5-fluorouracil (5-FU) with or without Oncorine at 5e11 to 1.5e12 VP/day for five consecutive days in between 2- and 43-week cycles. The response rates of patients with Oncorine plus chemotherapy and receiving chemotherapy alone were 78.8 and 39.6% (15). High seroprevalence against several adenovirus serotypes (including the backbone of Oncorine, serotype 5) limits the ability to deliver Oncorine intravenously to treat highly metastatic disease (47, 48), so using lower seroprevalence or modified knob proteins is a better way to transport Oncorine. These adenoviral vectors are now in clinical trials to test their safety and efficacy following intravenous delivery. While oncolytic adenoviruses have been in development for over 20 years (14), Oncorine remains the only approved adenovirus for cancer treatment and must be in combination with chemotherapy.

#### Herpesvirus

HSV1 is a double-stranded DNA virus, and it is about 152 kb in length (49). Herpes was the first genetically engineered virus to combat cancer. According to research in 1991, HSV-dlspTK, a TK-deleted HSV-1, improved overall survival in a murine model of glioblastoma (50). Then with the development of researches concerned, in this field appeared the generation, preclinical, and clinical testing of novel HSV gamma34.5-deficient viruses, which lack both neurovirulence and the ability to inhibit the antiviral PKR response (51). Clinically evaluated gamma34.5-deficient viruses contain T-VEC (52), HSV1716 (Seprehvir) (53), G207 (54), and RP1, which were announced in clinical trials in November 2017. NV1020 retained a single copy of gamma34.5 and contained additional attenuating mutations to TK, UL24, UL55, and UL56 at the same time, which has also been tested in human patients (55). Besides, a naturally existing HSV mutant HF-10 that retains copies of gamma34.5 has been clinically tested in patients with breast, head, and neck cancers (56).

There have been many tests in patients about OVs deriving from engineered HSV1. According to a report, 16.3% of patients with melanoma were improved after intratumoral injection of talimogene laherparepvec (18). The effects were most effective in patients with stage IIIB, IIIC, IVM1a, or treatment-naive disease. Moreover, tumor regression can also present in distant non-injected lesions (57).

#### T-VEC

Talimogene laherparepvec was approved for the treatment of non-resectable metastatic melanoma by the US FDA in 2015 and then approved for locally advanced or metastatic cutaneous melanoma in Europe. As a recombinant human HSV-1, T-VEC is deleted for both copies of the HSV1 gamma34.5 and viral ICP47 that can accelerate the expression of US11 and encodes two copies of human granulocyte-macrophage colony-stimulating factor (GM-CSF) with the help of cytomegalovirus (CMV) promoters (58). T-VEC was approved for the treatment of cutaneous high-grade melanoma lesions by intratumoral injection and showed single-agent efficacy (18). Single-agent efficacy was also being applied for evaluating patients with liver, pancreatic, and advanced nervous system solid tumors, as well as the safety and efficacy of T-VEC alone or in combination with checkpoint inhibitors, chemotherapy, or radiation therapy in melanoma. According to an article published in 2017, late-stage melanoma patients treated with T-VEC and PD-1 inhibitor pembrolizumab achieved a satisfactory result (59). The combination of T-VEC and PD-1 inhibitor pembrolizumab can have better efficacy and fewer side effects at the same time, especially in uninjected visceral metastases, which had a 7% response rate with T-VEC alone (18). Comparing the treatment of ipilimumab alone and combining anti-CTLA4 antibody ipilimumab with T-VEC, the result showed that the former treatment has a significant improvement in progression-free survival (PFS) of visceral metastases from 0% PFS to 23% PFS (60).

#### Adenovirus

Adenoviruses are non-enveloped icosahedral double-stranded DNA viruses, and each capsid vertex has long fiber knobs (61). There are currently at least 70 serotypes of human adenovirus, and serotype 5 is the most frequently used (six of seven oncolytic adenoviruses used in clinical trials was a serotype five backbone). Clinical data of concern have been published, including telomelysin in solid tumors (62), CG0070 in bladder cancer (63), and DNX-2401 in malignant brain tumors (64).

The binding of the adenovirus receptor appears at both RGD motifs of penton base proteins and fiber knobs that extend from them (65). Receptor specificity is dependent on virus subgroup and serotype, and there are at least 11 receptors that have been demonstrated to function in adenovirus binding (66). Many adenoviruses combine with integrins through penton RGD motifs, facilitating entry and infection of permissive cells (67). As a subgroup C virus, Ad5 also infects cells with the help of coxsackie adenovirus receptor (CAR), heparan sulfate glycosaminoglycans (HS-GAG), and some other receptors such as MHC-I, VCAM-1, and DPPC, while Ad3, a subgroup B virus, binds CD46, CD80, and CD86 (68). Modifications to the penton base RGD binding domain and serotype switching or modifications of fiber knob proteins are all trying to modify tissue tropism (69). There are many examples like the RGD-4C motif used in DNX-2401, which binds cell adhesion molecules and allows entry through any fibronectin-binding integrin receptor (70); the chimeric ONCOS-102 and LOAd703 viruses, which respectively, incorporate CD46-tropic serotype 3 and 35 fiber knobs into serotype five backbones (71); and inclusion of an RGDK motif in the HS-GAG binding domain of the fiber shaft of VCN-01, which detargets the virus from the liver and enhances tumor selectivity *in vivo* (72, 73).

Adenovirus is one of the most commonly used OVs to fight cancer. Among them, an adenovirus called E1A/E1B-deleted virus, named H101, has been widely used in the treatment of head and neck cancers in China (74). Compared with traditional radiotherapy and chemotherapy, this treatment has less toxic side effects and significantly improves patients’ quality of life at the same time.

#### Vaccinia Virus

Vaccinia is a giant, enveloped, double-stranded DNA virus with a linear genome approximately 190 kb in length (75). Up to now, three oncolytic vaccinia viruses are used clinically, isolated from Wyeth (SillaJen, JX-594, pexastimogene devacirepvec/Pexa-Vec), Western Reserve (Transgene, TG6002), and Lister (GeneLux, GL-ONC1/GLV-1h68) vaccinia strains. As a representative of the vaccinia virus, Pexa-Vec is engineered to express human GM-CSF and has been tested in more than 300 patients. It shows good results in the improvement of patients’ tolerance and prolonging the patients’ life (76). It is believed that the vaccinia virus has excellent potential in antitumor field.

#### Coxsackievirus

As a single-stranded positive RNA picornavirus of approximately 7.4 kb, Coxsackievirus is surrounded by an icosahedral capsid. Deriving from the Kuykendall strain, oncolytic CVA21 uses ICAM-1 as the primary receptor for cell entry (77). Some tests have been carried out in intratumoral or intravenous administration, a single agent or combination with immune checkpoint blockade, in several phase I/II clinical trials in patients with breast cancer, prostate cancer, bladder cancer, melanoma, and non-small cell lung cancer (NSCLC) (78).

A clinical trial about Coxsackievirus named Cavatak is ongoing, and numerous trials are carried out and based on solid 2015 phase 2 data in stage IIIC and stage IV melanoma. According to a report, the preliminary DRR is 21% as the regression of distant non-injected lesions (79).

#### Retrovirus

Retroviral replicating vector (Tocagen, Toca-511, vocimagene amiretrorepvec) encodes yeast cytosine deaminase (CD) that transforms the prodrug 5-FC into the anticancer drug that can increase the local concentration of 5-FU in the tumor and decrease overall systemic toxicity of the drug. Different from the OVs discussed above, these vectors are non-lytic but, instead, selectively replicate in dividing cells with defective innate immunity and interferon responsiveness (80).

About the clinical trial of the retrovirus, it is high profile that Toca 511 is currently in a phase 2/3 clinical trial for malignant glioma and showed positive medium-term results (81). Furthermore, retrovirus can probably be transformed into a powerful “weapon” to cure some malignant tumors, especially glioma.

#### Vesicular Stomatitis Virus

The selectivity of the VSV derives from the deficiency of interferon signaling (82). At present, the research on VSV is mainly about the treatment of liver cancer. As a case, an engineered VSV variant that overexpresses interferon β is in a clinical trial for liver cancer (63).

## Anticancer Mechanism of Oncolytic Virus

As promising cancer gene therapy agents, OVs have the unique ability to selectively replicate in cancer cells and cause the inflammation and even death of cancer cells, further leading to host immune responses because of cancer-associated antigen exposure (83). As is shown in Figure 1, the anticancer mechanism of the OV includes direct oncolysis or cytotoxicity toward the cancer cells or indirect induction of bystander effects (including the destruction of tumor blood vessels) and immunotherapeutic toward tumors (5, 84).

**FIGURE 1:** Anticancer mechanism of oncolytic virus.

After infection, the viruses can hijack the tumor cell’s protein factory and prevent tumor cells from producing enough protein to meet growth needs, thus destroying the normal physiological process of tumor cells. Besides, tumor cells can also be killed through the induction of immune response. Infected tumor cells can produce cytokines or chemokines, release tumor-derived antigens after apoptosis, and then attract a collection of immune cells including cytotoxic T lymphocytes, natural killer cells, dendritic cells, and phagocytic cells, which induce a tumor-specific immune response and potentially resulting in the elimination of uninfected cancer cells (85, 86). Eventually, it is worth noting that the immune response associates with an “immune-associated” bystander effect, in which local release of cytokines may cause the immune responses of nearby tumor cells, even without direct antigen expression (87). Except for the ones above, OVs can also destroy tumor blood vessels, reducing or even disrupting tumor blood supply, leading to tumor hypoxia and lack of nutrients (88, 89).

The necrosis induced by OVs can also cause the release of damage-associated molecular patterns (DAMPs), which stimulate dendritic cells and acquired immune responses (90). Besides, tumors can be divided into immunologically “cold” tumors and immunologically “hot” tumors according to the level of tumor antigen, CD8^+^ T cells, and immune-suppressive cells or cytokines (91). Although oncolytic virotherapy could kill cancer cells through direct oncolysis and activation of the immune response, the tumor can hinder antitumor immune response by interfering almost every step of immune activation and acquiring an immune-suppressive tumor microenvironment (92, 93). The OV can destroy the immune-suppressive environment through arming with immune-modulating genes including genes encoding inhibitors of immune checkpoints, tumor antigens, and targets for chimeric antigen receptor T cells, to further improve overall immune responses especially for immunologically “cold” tumors (94). However, solid tumors are complex, heterogeneous structures that hinder the oncolytic function of OVs. OVs can be engineered to increase their oncolytic ability by expressing modulatory molecules that target the structure of the tumor microenvironment to destroy tumor cells and impair the support for the growth of the tumor. Besides, the combination of OVs and immunostimulatory molecules can promote the development of antitumor immune responses. T-VEC, which was approved by the US FDA, recently can express granulocyte-macrophage colony-stimulating factor (GM-CSF) to treat melanoma (95). Treatment of advanced melanoma with T-VEC was safe and resulted in a 10.8% complete response rate, which was significantly higher than the systemic administration of GM-CSF alone (18). Thus, oncolytic virotherapy represents a new period of promising cancer virotherapy candidates.

Currently, the two most challenging problems of oncolytic virotherapy are as follows: (i) to ensure that the virus can maximize the ability of invasion and replication in tumor cells without infecting healthy tissues and cells to minimize the damage to the body and (ii) to prevent the virus from being eliminated by the body’s strong immune system, which leads to a significant reduction in the efficacy. For these two problems, on the one hand, the specificity of the OV can be enhanced by further modification of the genome; on the other hand, an attempt can be made to construct appropriate cell vectors for the OV. Healthy cells of the body can be selected to help the OV achieve immune evasion. On this basis, targeted drug therapy can combine with oncolytic virotherapy to enable OV-carrying targeted drugs in a certain way, thus enhancing the anticancer effect. It is believed that the future development direction of oncolytic virotherapy will be an organic combination of gene modifications, construction of virus carriers, and targeted drug therapy.

## Combination of Cancer Treatment Strategies With Oncolytic Virotherapy

### Tumor Targeted Cell Delivery Therapeutic Oncolytic Virus

Oncolytic virus therapy is a specific antitumor therapy, but the blood system is a very defensive environment in which innate and adaptive immune can neutralize virus particles and significantly decrease the efficacy (96). Therefore, it is urgent to find appropriate carriers to deliver the OV to tumor tissues for effective treatment. Carrier cell research is moving toward using cells that not only provide shielding from antibodies and complement but also detarget from off-target organs, home to tumor sites, and exert their antitumor effector functions. At present, the most commonly used cell carriers are cell carriers including antigen-specific T cell (AST), cytokine-induced killer cell (CIK), mesenchymal stem cells, and blood outgrowth endothelial cells (BOECs) (97–99). An optimal cell carrier must include the following characteristics: first, it must be susceptible to virus’ infection; second, it can assist the virus in locating the tumor tissue while not being recognized by the immune system; finally, it has the ability to release progeny virus to attack distant cancer cells (100). The specific anticancer mechanism of AST is that under the impact of chemokines, AST arrives at the tumor site, first through the surface adhesion molecule non-specific combination with tumor cells. Then the AST receptor combines with tumor surface-specific antigen-major histocompatibility complex and secretes tumor destruction factor, thus specifically killing tumor cells (101). In the case of CIK, CIK recognizes tumor cells by binding the NKG2D receptor with NKG2D ligand on the tumor surface. In a variety of disease models, non-invasive imaging techniques have shown that CIK infected with vaccinia virus can deliver vaccinia virus to tumor sites after intravenous injection and show strong antitumor effect. According to research, viral delivery to tumor tissue is more efficient using CIK carrier cells than the virus alone. What is more, the CIK carrier cells still retain their ability to exert antitumor destruction (102–104). Furthermore, this approach produces efficient tumor clearance in multiple cancer models so that CIK can be used as a cell carrier targeting tumor cells. In a study by Manish R. Patel, blood outgrowth endothelial cells were used to deliver VSV expressing IFNβ to metastatic NSCLC in mouse models. The result demonstrated that blood outgrowth endothelial cells could transport the OV efficiently and had great potential in clinical translation (105). As an efficient approach of virus delivery, the ultrasound-targeted microbubble destruction (UTMD) can help the OV to successfully pass the liver system and avoid the immune system’s clearance. In a study by Rupesh Dash, the UTMD was used to transport the therapeutic virus to the tumor site in mouse model of prostate cancer and obtained satisfactory experimental results (106). Besides, the emergence of a nanocarrier has attracted great attention. The nanocarriers with a higher delivery efficiency include lipid nanocarriers, polymeric nanocarriers, organic nanocarriers, and metal nanocarriers. They can enhance the OVs’ ability to increase concentrations of therapeutics at tumor sites, tumor selectivity and targeting, and hiding from the immune response (107).

### Genetically Engineered Oncolytic Virus

Also, to enhance the therapeutic effect, modifications in OVs through genetic engineering, including insertions and deletions in the genome, can deliver additional therapeutic molecules to cancer cells and effectively avoid the widespread resistance of single-target anticancer drugs (8). At present, there are nearly a hundred therapeutic exogenous genes in research, such as cell death-related molecules, anti-angiogenic molecules, and small RNA molecules (including miRNA, siRNA, shRNA, and lncRNA) that inhibit tumor-related genes. It is well known that the resistance to oncolytic virotherapy of tumor is related to the overexpression of PD-L1 expression on tumor cells and immune cells (108). In a study by Guan Wang, an OV that expressed PD-L1 inhibitor and GM-CSF was generated by genetic engineering technology. The PD-L1 secreted by the engineered OV could block PD-L1 on tumor cells and immune cells. The result showed that the OV could enhance the activity of cancer neoantigen-specific T cell responses and acquire more effective antitumor effects, especially for cancer patients insensitive to PD-1/PD-L1 blockade therapy (109). Besides, an OV armed with IL-7, IL-12, and IL-24 (110, 111) master pro-inflammatory cytokine interleukin 12 or Beclin-1 was all proved to have a superior antitumor activity than the parent OV (112–115). Suicide gene therapy is also one of the methods of tumor gene therapy, also known as viral-mediated enzyme hydrolytic drug precursor therapy (VDEPT). So-called suicide gene therapy is the introduction of a gene encoding a sensitive factor into tumor cells, so that the cells have a specific sensitivity to a non-toxic or low-toxicity drug, resulting in the death of tumor cells. In a study by Su-Nam Jeong, researchers constructed a novel oncolytic vaccinia virus by replacing the vaccinia growth factor (VGF) and viral TK (vTk) genes with genes expressing TNF-related apoptosis-inducing ligand (TRAIL) and angiopoietin 1 (Ang 1). This gene transition could enhance the ability of tumor-targeted apoptosis and immune response of the novel oncolytic vaccinia virus with high biosafety (116). Different from other combined therapies, the OV can achieve specific local expression effects through being armed with therapeutic transgenes, which, to a certain extent, means more accurate tumor killing. Besides, direct modification of foreign genes on reproducible OVs can obtain a long-term expression effect of related genes.

Due to the heterogeneity of tumor cells, it is unlikely to achieve a satisfying effect to treat tumors with monotherapy. Therefore, the combination of OV therapy and other therapies may be a better way to improve the efficacy and maximize the survival of patients.

### Combination of Radiotherapy With Oncolytic Viral Therapy

The combination of radiotherapy and oncolytic virotherapy has a synergistic effect on tumor treatment in multiple models (117–120). In one case, the synergistic effect between radiotherapy and virotherapy was observed with oncolytic HSV (121–125). The critical processes in this study are radiation-induced GADD34, the enhancement of viral promoters by p38, and oHSV-mediated inhibition of DNA repair (126, 127). Besides, radiotherapy can also be combined with oncolytic vaccinia virus to improve efficacy. One study showed that the synergistic effect depended on the inhibition of JNK signals induced by radiation (128). Moreover, VACV-scAb-VEGF was able to increase the sensitivity of tumor sites to radiation therapy. In a study using mouse xenografts as a model, VACV-scAb-VEGF increased the antitumor effect (129). Radiation therapy combined with oncolytic virotherapy can produce enhanced antitumor effects (130).

### Combination of Chemotherapy With Oncolytic Viral Therapy

There have been precedents of standard chemotherapy combined with virotherapy. For example, adenovirus has successfully combined with cisplatin, 5-FU, doxorubicin, temozolomide, irinotecan, and paclitaxel. The combination showed enhanced antitumor effects (131–134). At the same time, such combination therapy also showed higher safety, further extending the patient’s survival (135). Besides, the combination of vaccinia virus and paclitaxel also showed a synergistic effect. The mechanism is that paclitaxel enables cells to enter the s phase of the cell cycle, during which vaccinia virus is more likely to infect cells (136). In xenograft models, sorafenib combined with oncolytic vaccinia virus showed good antitumor results, while trials in patients show excellent safety and clinical response, and it has been approved for systemic use in liver, kidney, and thyroid cancers (137).

### Combination of Immune Checkpoint Inhibitors With Oncolytic Viral Therapy

Although there are few reports on the combination of immune checkpoint inhibitors and oncolytic virotherapy, immune checkpoint inhibitors targeting PD-1 or/and CTLA-4 combined with oncolytic virotherapy offers a new prospect for the treatment of cancer. Checkpoint inhibitors have synergistic effects with OV therapy in initiating or enhancing the immune response (138, 139). Several related studies have been conducted, and the results showed that OVs had more potent antitumor effects when combined with immune checkpoint inhibitors (140, 141). What is more, unpublished studies showed that the combination of immune checkpoint inhibitors and oncolytic virotherapy does not increase the side effects. It is expected that more immune checkpoint inhibitors can be found to combine with OVs for better treatment effect.

## Conclusion

Although many clinical trials about oncolytic virotherapy have confirmed the excellent treatment effect of oncolytic virotherapy, the therapy has some limitations. First, oncolytic virotherapy does not have a stable curative effect in different individuals because everyone’s physical environment is not the same, and OVs are too easy to be cleaned by the body’s immune system. Second, the biosafety of oncolytic virotherapy deserves further research, especially for people with low immunity. Third, the types of OVs currently available for clinical treatment or trail are limited. In order to deal with these problems and further improve the therapeutic efficacy of oncolytic virotherapy, we can combine the use of OVs, cell carrier construction, and tumor-killing drugs or molecule carried by OVs through genetic engineering organically, to achieve the best therapeutic effect and further extend the survival period of patients. Besides, more clinical trials are needed to ensure the biosafety of the oncolytic virotherapy, and more OVs should be constructed to be applied to clinical treatment as soon as possible. Moreover, it is believed that with the breakthrough of related research, oncolytic virotherapy will be popularized to the treatment of cancer soon.

## Author Contributions

G-DC and X-BH: writing of original manuscript. QS, S-HC, P-PL, BC, and M-MX: revision of the manuscript. KW, XX, and X-DF: language modification of the manuscript.

## Conflict of Interest

The authors declare that the research was conducted in the absence of any commercial or financial relationships that could be construed as a potential conflict of interest.
